This article has been retracted.

# Mouse-Induced Pluripotent Stem Cells Differentiate into Odontoblast-Like Cells with Induction of Altered Adhesive and Migratory Phenotype of Integrin

**DOI:** 10.1371/journal.pone.0080026

**Published:** 2013-11-11

**Authors:** Nobuaki Ozeki, Makio Mogi, Rie Kawai, Hideyuki Yamaguchi, Taiki Hiyama, Kazuhiko Nakata, Hiroshi Nakamura

**Affiliations:** 1 Department of Endodontics, School of Dentistry, Aichi Gakuin University, Nagoya, Aichi, Japan; 2 Department of Medicinal Biochemistry, School of Pharmacy, Aichi Gakuin University, Nagoya, Aichi, Japan; University of Newcastle upon Tyne, United Kingdom

## Abstract

Methods for differentiating induced pluripotent stem (iPS) cells into odontoblasts generally require epithelial–mesenchymal interactions. Here, we sought to characterize the cells produced by a ‘hanging drop’ technique for differentiating mouse iPS cells into odontoblast-like cells that requires no such interaction. Cells were cultured by the hanging drop method on a collagen type-I (Col-I) scaffold (CS) combined with bone morphogenetic protein (BMP)-4 (CS/BMP-4) without an epithelial–mesenchymal interaction. We evaluated the expression of odontoblast-related mRNA and protein, and the proliferation rate of these cells using reverse-transcription polymerase chain reaction, immunofluorescence staining, and BrdU cell proliferation enzyme-linked immunosorbent assay, respectively. The differentiated cells strongly expressed the mRNA for dentin sialophosphoprotein (DSPP) and dentin matrix protein-1 (Dmp-1), which are markers of mature odontoblasts. Osteopontin and osteocalcin were not expressed in the differentiated cells, demonstrating that the differentiated iPS cells bore little resemblance to osteoblasts. Instead, they acquired odontoblast-specific properties, including the adoption of an odontoblastic phenotype, typified by high alkaline phosphatase (ALP) activity and calcification capacity. The cell-surface expression of proteins such as integrins α2, α6, αV and αVβ3 was rapidly up-regulated. Interestingly, antibodies and siRNAs against integrin α2 suppressed the expression of DSPP and Dmp-1, reduced the activity of ALP and blocked calcification, suggesting that integrin α2 in iPS cells mediates their differentiation into odontoblast-like cells. The adhesion of these cells to fibronectin and Col-I, and their migration on these substrata, was significantly increased following differentiation into odontoblast-like cells. Thus, we have demonstrated that integrin α2 is involved in the differentiation of mouse iPS cells into odontoblast-like cells using the hanging drop culture method, and that these cells have the appropriate physiological and functional characteristics to act as odontoblasts in tissue engineering and regenerative therapies for the treatment of dentin and/or dental pulp damage.

## Introduction

Induced pluripotent stem (iPS) cells, in which non-pluripotent or somatic cells are forced back to a pluripotent state by the expression of specific genes, have great potential for cell transplantation-based regenerative medicine [1-3]. They also constitute a new tool with which to investigate organ differentiation in dental tissue. The development of dentin- or pulp-regeneration therapies involving human iPS cell-derived odontoblasts is a realistic aspiration for dentists aiming to treat patients that have suffered a loss of dentin or dental pulp tissue. There is ample evidence from the field of tooth development to implicate the molecular signaling pathways that drive odontoblast differentiation [4-6]. However, despite the potential of iPS cells in regenerative dentistry, their ability to differentiate into odontoblastic cells has not yet been investigated.

Bone morphogenetic proteins (BMPs), originally identified as protein regulators involved in embryogenesis and morphogenesis in various tissues including teeth [7,8], play an important role in dentin regeneration [9-11]. Specifically, dentin extracts induce the differentiation of dental pulp stem cells into cells that are capable of inducing dentin regeneration [7,12]. Although BMP-2 induces embryonic stem (ES) cells to differentiate into osteoblastic cells [13], it is possible that other BMPs might drive iPS cells to differentiate into odontoblastic cells. Characterization of the differentiated phenotypes of cells exposed to the various BMPs would give important clues as to which signaling systems are responsible for the differentiation of iPS cells into odontoblast-like cells.

The extracellular matrix (ECM) surrounding stem cells is unique to each type of tissue and not only provides a scaffold for support and organization but also generates the signals needed for survival, proliferation, and differentiation of these cells [14,15]. These structural proteins contribute to the unique properties that define the stem cell ‘niche’ for each tissue type and help maintain stem cell function and specification [15]. Furthermore, Nagai et al. demonstrated that the use of a collagen type-I (Col-I) scaffold for the differentiation of iPS cells could suppress the risk of teratoma formation [16]. Therefore, a Col-I-scaffold (CS) appears to be an effective device for investigating the odontoblastic differentiation of iPS cells.

We previously established a method for inducing isolated integrin α7-positive human skeletal muscle stem cells to undergo myogenesis and adopt the phenotypes of other mesenchymal cell such as osteoblasts and adipocytes [17]. Furthermore, a method for the differentiation of ES cells into neural-crest cells and odontoblast-like cells was previously reported [18], but this requires an epithelial–mesenchymal interaction. No method for differentiating iPS cells into odontoblastic cells without this interaction has yet been reported. Therefore, in the present study, we examined whether iPS cells could differentiate into odontoblast-like cells when cultured on a CS combined with BMP-4 (CS/BMP-4) and retinoic acid (RA). We optimized the culture conditions for achieving odontoblastic differentiation from mouse iPS cells, and thus acquired odontoblast-like cells that may be useful tools in novel tooth regenerative therapies.

## Materials and Methods

### Cells and culture

The mouse iPS cell line iPS-MEF-Ng-20D-17 was kindly donated by Prof. Yamanaka (Kyoto, Japan) and maintained as previously described [1,3]. The E14Tg2a ES cell line [19,20] (a kind gift from Dr. Randall H Kramer (University of California, San Francisco, CA, USA)) and the rat odontoblast-like cells (KN-3; kindly provided by Dr. Chiaki Kitamura, Kyushu Dental College, Kitakyushu, Japan) were maintained as previously described [21]. Mouse osteoblast-like MC3T3-E1 cells were from the Riken cell bank and cultured as previously described [22-24].

### Odontoblastic differentiation

The protocol for embryoid body (EB) formation from iPS cells was based on a published method for differentiating ES cells [25]. Purified odontoblast-like cells derived from ES cells were prepared by reported previously [26]. Cell aggregates were pooled on non-adherent culture dishes (Sumilon; Sumitomo Bakelite Co., Ltd., Tokyo, Japan) and cultured in suspension with 1×10^-7^ mol/L RA (Sigma-Aldrich, St. Louis, MO, USA) for 3 days to form neural-crest cells. These neural-crest cells (1.5×10^5^ cells/cm^2^) were then transferred to a CS, which consisted of a Transwell^®^ cell culture insert (8 μm pore size, PET track-etched membrane; Becton Dickinson Labware, Franklin Lakes, NJ, USA) with 10% collagen type-I (Col-I; PureCol collagen; Biomaterials, Fremont, CA, USA) coated onto the upper chamber. This coated upper chamber was then filled with serum-free Dulbecco’s modified Eagle’s medium (DMEM; Invitrogen, CA, USA), while the lower chamber was filled with differentiation medium consisting of DMEM (Invitrogen), 15% fetal bovine serum (Invitrogen), and BMP-4 (100 ng/mL; Peprotech Inc., Rocky Hill, NJ, USA) (Figure 1). Cells were incubated for 7 days in this differentiation medium to induce the iPS-derived EB cells to differentiate into odontoblast-like cells. Cultures were maintained at 37°C in a 5% CO_2_ humidified incubator, and the medium was changed every 2 days. Finally, the cells that had migrated into the lower chamber were detached and harvested with 3 mM EDTA in PBS. This experimental protocol is depicted in Figure 1.

**Figure 1:** Schematic representation of the experimental protocol used for odontoblast differentiation of mouse iPS cells. EB, embryoid body; RA, retinoic acid; CS: collagen type-I scaffold.

### Cell proliferation assay

Cell proliferation was evaluated using the BrdU cell proliferation ELISA (Roche Applied Science, Mannheim, Germany) as previously described [22-24], using cells seeded in 96-well tissue culture plates at a density of 1×10^5^ cells/cm^2^.

### Functional assay for assessment of the odontoblastic phenotype

To assess the phenotype of the cultured cells, we measured alkaline phosphatase (ALP) activity (as a marker of differentiation) and calcification. ALP activity was determined using an ALP Staining Kit (Primary Cell Co., Ltd., Hokkaido, Japan). Mineralization from the embryonic stem cell-derived odontogenic cells was quantified using the Alizarin red S (ARS) assay (Sigma-Aldrich). ARS staining was quantified using a method reported previously by Gregory and colleagues [27], and observed and photographed using a BZ-9000 microscope (Keyence, Osaka, Japan).

### Reverse-transcription polymerase chain reaction (RT-PCR)

The protocol for RT-PCR was described previously [17]. The PCR reaction within the exponential phase of the amplification curve was performed for 25 cycles for DSPP, Dmp-1, and Runx-2 (as odontoblast markers); Nanog, and SSEA-1 (as markers of undifferentiated cells); FoxD3 and Sox10 (as neural-crest markers); osteopontin and osteocalcin (as osteoblast markers); α-fetoprotein (AFP) and cancer antigen 125 (CA125) (as teratoma-specific genes); and GAPDH (as a housekeeping gene). The sequences of the gene-specific primers synthesized by Sigma-Aldrich are listed in Table 1. The PCR reaction was performed in a thermal cycler (GeneAmp PCR System 9700; Applied Biosystems, Carlsbad, CA, USA) using the following protocols: initial denaturation for 2 min at 94°C (all markers); denaturation for 30 s at 94°C (all markers); annealing for 30 s at 67°C (for mouse Nanog, mouse and rat DSPP, and mouse Dmp-1), 68°C (for mouse SSEA-1, mouse FoxD3, mouse Sox10, mouse osteopontin, and mouse osteocalcin), 64°C (for mouse GAPDH), or 61°C (for rat GAPDH); and extension for 1 min at 72°C (all markers). The PCR products were loaded onto a 1.5% agarose gel, electrophoresed, visualized with ethidium bromide under ultraviolet light and photographed. The relative intensities of the PCR products were quantified using a Multi Gauge-Ver3.X (Fujifilm, Tokyo, Japan).

**Table 1:** Primers for RT-PCR.

**Gene**	**Sequence**	**Product size (bp)**	**Accession number**	**Species**
Nanog	aggaagcatcgaattctgggaac tgaagaggcaggtcttcagagg	145	NM_028016	Mouse
SSEA-1	ccaggagggagcagtgacg gaatcgccctcccatactcca	109	NM_010242	Mouse
DSPP	cggaggctttgaagacattgattac gcagttcctggatgtgttagaagag	165	NM_010080	Mouse
Dmp-1	ctgtgctctcccagttgcca ggtcactatttgcctgtccctct	152	NM_016779	Mouse
FoxD3	cgacgggctggaggagaag ggcttgcggttgagaactgg	130	NM_010425	Mouse
Sox10	gagtgcccacctggaccac tctgccttgccggactgc	141	NM_011437	Mouse
Runx-2	ctccaccacgccgctgtc agggatgaaatgcttgggaactg	198	NM_001146038	Mouse
Osteopontin	ggtgcctgacccatctcaga tggaattgcttggaagagtttcttg	104	NM_001204201	Mouse
Osteocalcin	acacagcagcttggcccag gggcttggcatctgtgaggt	108	NM_007541	Mouse
AFP	ccctacagaccatgaaacaagagc tttggaaatcaactttggaccctc	176	NM_007423	Mouse
CA125	caccaaataccagcaaaccaaaaga gttgttgttggagacagacctgaa	127	XM_911929	Mouse
GAPDH	aatggtgaaggtcggtgtgaac cgtgagtggagtcggaac	155	NM_008084	Rat
Nanog	aacctgagctataagcaggtgaag cgctgagcccttctgagtca	117	NM_001100781	Rat
SSEA-1	acgcaccgaatgaggctctg cacacccaccgctgaccc	117	NM_022219	Rat
DSPP	tgcattttgaagtgtctcgc cctcctgtcttggtgtggtt	171	NM_012790	Rat
Dmp-1	cctgtgctcccctgtcgc ccgtgtggtcactatttgccat	114	NM_203493	Rat
FoxD3	cgatgtggtgggcgaggg agggcgttgaggttgagactgg	153	XM_575873	Rat
Sox10	cggcacccagaagaaggctc ggtggttggaggggtaggag	90	NM_019193	Rat
Runx-2	ccagatgggactgtggttac acttggtgcagagttcaggg	381	NM_053470	Rat
Osteopontin	gctcagaggagaaggcgcatta ttggagttgcttggaagagtttct	160	NM_012881	Rat
Osteocalcin	ctctgacctggcaggtgcaa gggctggggctccaagtc	128	NM_013414	Rat
GAPDH	actcccattcttccacctttg tgtagccatattcattgtcatacc	96	NM_017008	Rat

### Immunofluorescence microscopy

Immunofluorescence staining was performed as previously described [28]. Cells were seeded at 1×10^4^ cells per well on chamber slides (Nalge Nunc Int., Rochester, NY, USA) coated with poly-L-lysine (Sigma-Aldrich) and cultured overnight. After fixing with 1% paraformaldehyde for 15 min, cells were permeabilized with methanol at -20°C for 10 min. Non-specific binding was blocked by incubating cells with 10% normal goat or rabbit serum (Invitrogen-Gibco) in PBS for 1 h. Next, primary antibody against dentin sialoprotein (DSP; 2μg/ml; sc-18328; Santa Cruz Biotechnology Inc., Santa Cruz, CA, USA) was added in 1% normal goat serum for 1 h. Finally, cells were stained with fluorescein isothiocyanate (FITC)-labeled anti-goat IgG secondary antibody (Jackson ImmunoResearch Laboratories Inc., West Grove, PA, USA) for 30 min and cell nuclei visualized with 4',6-diamidino-2-phenylindole (Invitrogen-Gibco). Stained samples were imaged with a BZ-9000 microscope (Keyence). In preliminary experiments, we confirmed that these antibodies exhibited no significant cross-reactivity with other proteins (data not shown). No immunoreactivity was observed with control IgG.

### Flow cytometry

Flow cytometry was conducted using standard procedures [17,29]. Cells (1×10^6^ per ml) were incubated with predetermined optimal concentrations of primary antibodies for 1 h at 4°C, then washed and incubated with FITC-conjugated secondary antibodies (affinity-purified goat anti-hamster or anti-rat antibodies; Jackson ImmunoResearch Laboratories Inc.). Cells were then labeled with propidium iodide (1 μg/mL; Sigma-Aldrich) for 1 h at 4°C and processed using a FACSCalibur (Becton, Dickinson and Co., Franklin Lakes, NJ, USA).

To detect mouse integrin proteins, we used monoclonal antibodies (mAbs), kindly provided by Dr. Randall H. Kramer (UCSF, USA), except where indicated. These mAbs were anti-mouse integrin β (Ha2/11), anti-mouse integrin α (Ha31/8), anti-mouse integrin α2 (Ha1/29), anti-mouse integrin α3 (clone 42; BD Biosciences, San Jose, CA USA), anti-mouse integrin α5 (6F4), anti-rat integrin α6 (GoH3; Santa Cruz Biotechnology Inc.), anti-mouse integrin α7 (Cy8), anti-mouse integrin αV (L230), and anti-mouse integrin αVβ3 (23C6; Santa Cruz Biotechnology Inc.). These antibodies exhibited no significant cross-reactivity with other proteins (data not shown). For surface marker analysis, data were typically collected from 10,000 cells and analyzed with CellQuest Pro 4.1 software (BD Biosciences, San Jose, CA, USA). Unstained cells and cells incubated with secondary antibody only were both used as negative controls; background staining was similar to that using the isotype-control antibody.

### Cell adhesion and migration assay

Analysis of cell adhesion was performed as described previously [17,29]. Single-cell suspensions were incubated for 20 min on fibronectin (Fn) (5 μg/mL; Chemicon, Temecula, CA, USA) or 30 min on Col-I (1 μg/mL) at 37°C. Cell migration was assayed as described previously [30]. The undersides of Transwell inserts (8 μm pore size; BD Biosciences) were pre-coated with Fn (5 μg/mL) or Col-I (1 μg/mL). Cells migrating through the filter were counted manually under observation through a 20× objective lens and averaged from 10 randomly chosen microscopic fields.

### Statistics

All data are expressed as the mean±standard deviation (SD). Statistical significance was assessed using the Mann–Whitney U-test. *P* values less than 0.05 (*P* < 0.05) were considered as statistically significant.

## Results and Discussion

### Effect of scaffold type on cell proliferation

We first addressed which ECM component (i.e., Col-I, gelatin, Fn or Col-IV) was the most suitable to support the proliferation of the iPS cells and their differentiation into odontoblast-like cells. The BrdU cell proliferation ELISA results showed us that Col-I was the most suitable ECM component (Figure 2A). Interestingly, similar results were obtained for the E14Tg2a ES cells (Figure 2B). We next tested the capacity of the Col-I scaffold (CS) to induce proliferation of EBs derived from iPS cells. Cells were cultured on Col-I substrates for 14 days and their cell proliferation evaluated by BrdU cell proliferation ELISA. We found that, of the concentrations tested, 10% collagen in the CS was optimal for proliferation (Figure 2C and D).

**Figure 2:** Optimization of ECM components required to differentiate iPS cells into odontoblast-like cells. To evaluate the effect of extracellular matrix (ECM) components on the proliferation of embryoid bodies derived from iPS (A) and E14Tg2a ES cells (B), we cultured these cells on various ECM proteins for 14 days, examining cell proliferation at various time points during this period using a BrdU-based cell proliferation ELISA. Data are the degree of cell proliferation normalized against the number of proliferating cells at the start of the assay period (fold of control). Statistically significant increases in proliferation are shown by * and ** (*P* < 0.05 and *P* < 0.01, respectively, *vs*. control). The optimal concentration of collagen scaffold was also determined by growing iPS (C) and E14Tg2a (D) cells for 14 days *in* *vitro* on plates pretreated with various concentrations of CS (3%, 5%, 7%, 10%, or 15% Col-I). Proliferation was measured at various time points using a BrdU-based ELISA, as above. Data are the mean ± SD of three independent repeats. Differences between untreated and the various CS-treated groups were assessed using a Mann-Whitney U-test (*P < 0.05; **P < 0.01, *vs*. untreated).

To assess their potential for odontoblast differentiation, we evaluated the response of iPS cells to BMP-2, -4, and -7. Following the differentiation protocol, samples were assessed by RT-PCR for differentiation markers. When EBs were cultured with 10% CS combined with BMP-2 (300 ng/mL), BMP-4 (100 ng/mL) or BMP-7 (100 ng/mL) for 7 days, only the BMP-4-treated cells showed higher mRNA expression of the odontoblast markers DSPP and Dmp-1 (data not shown). Therefore, BMP-4 (100 ng/mL) was chosen in the current system as an odontoblast differentiation factor.

Using these optimized experimental conditions, we found that after 5 days of culture, the EBs could be cultured on a CS with 10% Col-I and BMP-4 (100 ng/mL) to undergo odontogenic differentiation. Dentin sialophosphoprotein (DSPP) is cleaved immediately after secretion into two daughter proteins (DSP and dentin phosphoprotein) [4,31,32]. Since DSPP is highly expressed in odontoblasts, DSP is considered to be an odontoblast-related marker. Dentin matrix protein (Dmp-1) is also expressed by differentiating odontoblasts during development [33]. The expression of DSPP and Dmp-1 in functional odontoblasts in early stages of odontogenesis is consistent with the roles that both DSPP and Dmp-1 play in the mineralization of dentin [33,34]. To evaluate the odontoblastic potential of iPS cells, we performed immunofluorescence staining to detect DSP. The DSP-specific staining was very low in undifferentiated cells but increased markedly following odontoblast differentiation (Figure 3A-a,b). A similar result was obtained for E14Tg2a ES cells (Figure 3A-c,d), suggesting that the iPS cell-derived differentiated cells had acquired DSP as a relatively specific odontoblastic marker. On day 12, after 10 days of odontoblastic differentiation following EB formation, the differentiated iPS cells were observed to have spread outward with dendrite-like extensions from the attached EBs (Figure 3A-b).

**Figure 3:** Odontoblastic differentiation of iPS cells on CS/BMP-4. (A) Immunofluorescence staining for the odontoblastic cell marker, dentin sialoprotein (DSP). Images show iPS cells (a, b) and E14Tg2a cells (c, d) that are undifferentiated (a, c) or differentiated using CS/BMP-4 (b, d). Scale bars = 25 μm. (B) Odontoblastic-related mRNA expression in these differentiated cells. Cells were cultured for 7 days with 10% CS and BMP-4 and the expression of various markers (as shown) assessed by RT-PCR. Rat KN-3 odontoblast-like cells (c) were used as a positive control. Mouse MC3T3-E1 cells (d) were used as an osteoblastic control. Band densities for each cell type cultured in the absence (control: white bars) or presence (black bars) of CS/BMP-4 for 7 days were evaluated using a Multi Gauge-Ver3.X (Fujifilm, Tokyo, Japan). Data are normalized against the housekeeping gene, GAPDH, and are presented as the mean ± SD of at least three independent experiments.

### Expression of odontogenic-related mRNAs in the iPS cell-derived differentiated cells

Using RT-PCR, we investigated the transcription of odontoblast-like markers in iPS cells and E14Tg2a ES cells on day 0 (control) and day 12 of differentiation with CS/BMP-4 (Figure 3B-a and b). DSPP mRNA was detected on day 12 in differentiated iPS cells, but not at day 0. In contrast, the mRNA expression of the undifferentiated cell markers Nanog and SSEA-1 was lost in the differentiated iPS cells on day 12 compared with their expression on day 0 (Figure 3B-a). FoxD3 and Sox10 (neural-crest markers) and Dmp-1 and Runx-2 (mature odontogenic markers) in the differentiated iPS cells were also clearly induced on day 12, with an identical expression profile occurring in the differentiated E14Tg2a cells and odontoblast-like KN-3 cells (Figure 3B-b and c). Since the osteoblastic markers osteopontin and osteocalcin were not expressed in the differentiated iPS cells, we concluded that the iPS cells had differentiated into odontoblastic cells rather than osteoblastic ones (Figure 3B-a). Thus, the differentiated iPS cells expressed mRNAs encoding odontoblast-related molecules at comparable levels to those seen in the differentiated E14Tg2a cell line and KN-3 cells. These cells can thus be said to be odontoblastic.

Importantly, we also confirmed that CS was suitable for inducing the formation of odontoblasts from iPS cells without inducing the expression of teratoma-specific genes such as AFP and CA125 (Figure 3B-a). This is highly important when considering the use of such cells in human transplantation therapies.

### Odontoblast differentiation of iPS cells

Having characterized the genetic phenotype of the differentiated iPS cells, we aimed to assess their functional phenotype by measuring their ALP activity and calcification capacity (Figure 4A, B). The majority of CS/BMP-4 cells showed potent ALP expression, whereas control cells did not (Figure 4A). We next tested whether CS/BMP-4 could induce mineralization in the iPS cells and E14Tg2a cells, as evaluated by staining with ARS. We observed extensive deposits of calcified matrix in the CS/BMP-4 cells, which were not apparent in control cells (Figure 4B). Interestingly, as the odontoblastic cultures progressed, ALP activity increased (Figure 4A). In agreement with the results above, CS/BMP-4 treatment resulted in a strong increase in the ARS signal (Figure 4B). These data demonstrate that iPS- and E14Tg2a-derived cells acquire odontoblast-specific functions following differentiation, further confirming our conclusions from above that the iPS cell-derived differentiated cells appeared to be odontoblastic.

**Figure 4:** Expression of odontoblastic functional phenotypic markers. (A, B) Alkaline phosphatase (ALP) activity and calcification capacity are characteristic of differentiated odontoblasts, so were measured in iPS cells and E14Tg2a cells treated with or without CS/BMP-4. (A) ALP activity was measured by absorbance at 405 nm and normalized against total protein. (B) The mineralization of iPS and E14Tg2a cells was assessed by Alizarin Red-S (ARS) staining. ARS was measured as absorbance at 405 nm by an SH-1200 Lab instrument. Scale bars = 100 μm. (*P < 0.01, *vs*. control).

### Differentiation-induced changes in integrin expression profile

To test whether ECM-related cell-surface receptor proteins were expressed on these cells, we used flow cytometry analysis to measure changes in integrin expression following odontoblastic differentiation. As for undifferentiated iPS cells, we found low-level expression of a diverse set of integrin α chains (i.e., α1, α2, α3, α5, α6, α7, αV, and αVβ3 integrin) (Figure 5A). Following differentiation with the CS/BMP-4 treatment, there was a marked increase in the expression of integrin α2, α6, αV, and αVβ3 subunits (Figure 5A). The increase in the expression of integrin α2 was particularly notable. Similar results were obtained in the E14Tg2a ES cells (Figure 5B).

**Figure 5:** Flow cytometry analysis of integrin expression. Cells were cultured in the absence (control: grey bars) or presence (black bars) of CS (10% Col-I) and BMP-4 for 7 days in the presence of various anti-integrin monoclonal antibodies (as shown). Detection of the relevant secondary antibody was performed by flow cytometry to estimate the numbers of cells expressing each protein. Negative control values (secondary antibody alone) were subtracted from test values to give the mean fluorescence intensity. Data are mean ± SD (n=3).

### Expression of integrin α2 induced by odontoblastic differentiation

To examine whether the integrin expression by the CS/BMP-4 treatment was a key step in the differentiation of iPS cells into odontoblastic cells, we investigated the effects of adding anti-integrin α2 antibody during culture in the CS/BMP-4 setup, and found that this antibody suppressed the expression of the odontoblastic markers, DSPP and Dmp-1. In contrast, anti-α1, anti-α3, anti-α5, anti-α6, anti-α7, anti-αV, and anti-αVβ3 antibodies had no such effect (Figure 6A). Similar results were obtained in E14Tg2a ES cells (Figure 6A). Importantly, we confirmed that this effect was not due to cytotoxicity because the addition of anti-α2 integrin antibody to cultures for 7 days had no effects on cell attachment, proliferation, or cell death (data not shown). We thus concluded that the expression of α2 integrin in iPS cells was a trigger for differentiation into odontoblast-like cells.

**Figure 6:** Effect of anti-integrin antibodies and siRNA silencing on induction of odontoblastic markers. (A) The expression of odontoblastic marker mRNAs (DSPP and Dmp-1) in CS/BMP-4 differentiated iPS cells and in E14Tg2a odontoblastic cells was assessed by RT-PCR following culture in the presence of various anti-integrin monoclonal antibodies (5 μg/ml). No significant cross-reactivity with other integrin proteins was observed for these antibodies. Images shown are representative of at least three independent experiments. (B) The effect of transfection of iPS cells and E14Tg2a cells with an integrin α2-specific siRNA. Images show RT-PCR analysis of integrin α2 mRNA expression in cells 24 h after transfection with siRNA (top panels), with expression of the housekeeping gene, GAPDH, as a control (second panels). Western blot analysis (lower three panels) show integrin α2 protein expression in these cells 24 h after siRNA transfection. (C) As in B, iPS cells and E14Tg2a cells were treated with an integrin α2-specific siRNA and the expression of DSPP and Dmp-1 mRNA and protein were measured.

### Effect of siRNA silencing on integrin α2-induced odontoblastic differentiation

Cells were transfected with integrin α2 siRNA (or a negative control siRNA) and cultured as described above. RT-PCR and western blot analysis showed that expression of integrin α2 mRNA and protein was ablated in cells transfected with the integrin α2 siRNA (Figure 6B). In contrast, the negative control siRNA did not attenuate integrin α2 mRNA or protein. There was no change in the expression of the GAPDH housekeeping gene or β integrin protein following siRNA treatment, demonstrating the specificity of the siRNA knockdown. Second, we demonstrated that transfection of integrin α2 siRNA efficiently down-regulated the expression of DSPP and Dmp-1 (Figure 6C), whereas the control siRNA did not. Finally, when we investigated the induction of ALP activity as an odontoblast marker, and found that the majority of ALP activity was lost when cells were pretreated with the integrin α2 siRNA (Figure 7). Similarly, we tested whether integrin α2 siRNA affected the mineralization capacity of the iPS cell-derived odontoblast-like cells by staining with ARS and found that the integrin α2 siRNA ablated the extensive deposition of matrix in the CS/BMP-4-treated cells (Figure 8). Similar results were obtained when blocking integrin α2 (Figure 7 and Figure 8). These data confirm that the expression of integrin α2 is required for the emergence of odontoblast-specific functions in differentiated iPS cells.

**Figure 7:** Effect of anti-integrin α2 mAb and siRNA on functional activity in odontoblast-like cells. Effect on ALP activity. CS/BMP-4-differentiated iPS cells and E14Tg2a cells were treated with either integrin α2-specific siRNA (or control siRNA) or anti-integrin α2 mAbs (or control mAbs). ALP activity data are presented as the mean ± SD (n=4) of the absorbance at 405 nm, normalized against total protein.

**Figure 8:** Effect of anti-integrin α2 mAb and siRNA on mineralization capacity in odontoblast-like cells. Cells were prepared as in A and cell mineralization was assessed by Alizarin Red-S (ARS) staining, with quantification performed by measuring absorbance at 405nm. Data are the mean ± SD (n=4). **P < 0.01, vs. control; *^#^P* < 0.01, as indicated by brackets.

As shown in Figure 6B, treatment with siRNA against α2 integrin could not suppress b1 integrin protein in odontoblasts derived from iPS and ES cells. β1 integrin is ubiquitously expressed and can bind to multiple partners, such as α1, α2, α4, α5, α6, α7, α8, α9, α10, α11, αV integrin, among others [35]. In contrast, b1 integrin is the only partner for α2 as seen in the α2β1 complex. As the interaction between the α integrin and the β integrin plays an important role in the physiological function of the complex, the knockout of β1 integrin would also be expected to generate a similar suppression of differentiation in current system due to an incomplete formation of α2β1 integrin complex. However, because of the ubiquitous distribution of the β1 integrin, we only chose to knock out α2 integrin to test the importance of the complex in these cells.

### Odontoblastic differentiation-induced changes in adhesion and motility

To examine whether the induced integrin expression equipped the cells with specific physiological functions, we assessed cell adhesion to Fn and Col-I substrata following CS/BMP-4-induced differentiation in the presence and absence of pre-optimized concentrations of integrin-blocking monoclonal antibodies. Whereas only a minor fraction of the undifferentiated iPS cells adhered to Fn, differentiation dramatically enhanced the ability of the iPS cells to adhere to this substratum (Figure 9A). This adhesion was specifically blocked by anti-αV, anti-αVβ3, and anti-β1 mAbs, suggesting the involvement of these integrins in cell adherence, in keeping with our earlier finding that integrin αV is strongly expressed in these differentiated cells (Figure 9A). Similarly, differentiation enhanced adhesion of iPS cells to Col-I substrate, which was disrupted by the anti-integrin α2 mAb (Figure 9B) and the anti-integrin β1 mAb.

**Figure 9:** Adhesion and motility of differentiated cells on collagen type-I and fibronectin. (A, B) The adhesion of differentiated (black bars) and undifferentiated (white bars) iPS cells to a substratum of either Fn (5 μg/ml; A) or Col-I (1 μg/ml; B) was assayed in the presence of the indicated anti-integrin antibodies. Data are the number of adherent cells, expressed as a percentage of the total number of cells. Bars indicate the standard deviation. (C, D) Similar experiments were used to investigate motility. The migration of differentiated (black bars) or undifferentiated cells (grey bars) through Transwell inserts coated with Fn (5 μg/ml; C) or Col-I (1 μg/ml; D) was assayed in the presence of the indicated anti-integrin antibodies. Cells were added to the upper chamber and incubated for 3 h. Motility was estimated by counting the number of cells that had migrated to the undersides of the membranes. Data presented are the mean ± SD of at least 10 random microscopic fields.

We also tested the ability of differentiated and undifferentiated cells to migrate on these same Fn and Col-I substrata. Because adhesion is a key stage in migration, it was not surprising that we obtained very similar results to the adhesion studies described above. Undifferentiated cells did not migrate on either substrate, whereas differentiation caused a dramatic increase in cell locomotion on both substrates (Figure 9C and D). Migration on Fn was blocked by mAbs against integrins αV, αVβ3 and β1 (Figure 9C), whereas that on Col-I was disrupted by anti-α2 and anti-β1 antibodies (Figure 9D). Nearly identical adhesion and motility results were observed for the ES cell lines (data not shown).

In summary, we have shown that iPS cells can be induced to differentiate without any need for epithelial–mesenchymal interactions using a novel hanging drop method that employs a collagen scaffold and BMP-4 as the differentiation matrix. This system produces convincingly odontoblastic cells that express odontoblastic markers at similar levels to true odontoblast cell lines, perform odontoblastic functions, and acquire odontoblast-like integrin expression profiles and adhesion and migration behaviors.

Odontoblast cells produced in bulk from iPS cells may represent an important source of dental cells for use in tissue engineering (e.g. regeneration and stem cell therapy). The goal of human transplantation mandates careful consideration of safety aspects, notably that the cells produced are not teratogenic. The CS is known to suppress the risk of teratoma in iPS-derived cells [16], but the novelty of our current method meant that we had to confirm that it also suppressed the expression of teratoma-related genes in the iPS cell-derived odontoblasts, which it did. Therefore, we are confident that these cells would be safe for human application.

The differentiation of iPS cells on the CS/BMP-4 matrix appears to be integrin-α2-dependent. Little is known about how extracellular signals induce differentiation, but the modulation of adhesion receptors may be an important mechanism by which stem and progenitor cells are recruited to target tissues. Importantly, interactions between the ECM and integrins on stem cells resident in a tissue microenvironment may be the specific cues required for terminal differentiation and tissue-specific regeneration. Integrin expression is also fundamental to adhesion and motility, which are vital functions in tissue remodeling and repair. It is interesting that the integrin expression profiles, adhesion and motility of the iPS-derived cells match those of odontoblast cell lines and cells derived from ES cells, as this suggests that these iPS-derived cells may have true functional potential in colonizing and repairing tooth tissues. However, the link between differentiation, integrin expression and cell adhesion in these cells remains to be fully elucidated and requires further investigation.

## Conclusions

The present study describes a highly novel cell culture method for producing odontoblast-like cells from mouse iPS cells, using a CS/BMP-4 matrix. The cells exhibit relevant physiological functionality and appear to be non-teratogenic. We conclude that this technique has great potential as a cell source for tissue engineering and regeneration of odontogenic tissue, producing cells capable of repairing dentin and possibly facilitating the re-establishment of lost dental pulp.
